The article "Dynamic connectedness and spillovers between Islamic and conventional stock markets: time- and frequency-domain approach in COVID-19 era" was retracted in 2025. Reasons: unreliable results or conclusions; concerns about the peer review.

# Dynamic connectedness and spillovers between Islamic and conventional stock markets: time- and frequency-domain approach in COVID-19 era

**DOI:** 10.1016/j.heliyon.2022.e09215

**Published:** 2022-03-31

**Authors:** Ahmed Bossman, Peterson Owusu Junior, Aviral Kumar Tiwari

**Affiliations:** a Department of Finance, School of Business, University of Cape Coast, Cape Coast, Ghana; b Rajagiri Business School, Rajagiri Valley Campus, Kochi, India

**Keywords:** Dynamic connectedness, Volatility spillovers, Conventional stock markets, Islamic stock markets, Time- and frequency-domain, COVID-19 pandemic, Contagion

## Abstract

This study investigates the dynamic connectedness and spillovers between Islamic and conventional stock markets to reveal the time- and frequency-domain dynamics of the two asset classes under various market conditions. Using the spillover index of Baruník and Křehlík (2018), supplemented by the time-varying parameter vector autoregressions (TVP-VAR) connectedness model, we employ daily stock market indices for Islamic and conventional (G7) markets from November 23, 2015, to September 8, 2021. The findings explicate that the volatility spillovers across and within Islamic and/or G7 markets are time-varying and frequency-dependent but during market turbulences, the conventional stocks are prone to more volatilities than the Islamic stocks. Our findings additionally divulge contagious spillovers among Islamic and conventional stocks during Brexit and the studied COVID-19 period. Relative to mid-and long-term spillovers, we underscore the supremacy of short-term spillovers between Islamic and G7 markets. In turbulent trading periods, investors should utilise knowledge about market patterns and volatility to hedge their positions against lower stock returns, when spillover is more intense. Regulators should pay close attention to spillovers since they undermine cross-market connections. Intriguing findings and their implications are further discussed.

## 1 Introduction

Islamic equities have grown in popularity in recent years, particularly after the global financial crisis (GFC) of 2008/09 and the European debt crisis (EDC) of 2011/12 (Bossman, 2021). Several studies (Balli et al., 2019; Shahzad et al., 2018; etc), have shown that Islamic equities outperform their conventional counterparts during times of financial crisis. Islamic stocks and indices have provided a popular channel for investors to incorporate their religious views into their investments. According to Ng et al. (2020), the Islamic Finance Development Indicator (IFDI) in 2018 showed that the durability of the Islamic financial market is demonstrated by its extraordinary development, evidenced by a growth rate of about 11% per annum, making it appealing to investors.

Lee and Goh (2016) observe a complete market integration across traditional financial markets, which limits portfolio diversification possibilities, making investors lose faith in conventional financial markets. Ng et al. (2020) opine that since investors have started to lose faith in traditional financial markets, Shariah-compliant stock is recognised as one of the main investment vehicles utilised in building optimum investment portfolios in Islamic financial markets (IFMs). When studies (Balli et al., 2019; Hassan et al., 2020; Hassan et al., 2020; Shahzad et al., 2018; etc.) discovered that Islamic stocks might satisfy investors’ risk tolerance or risk aversion, particularly during the global financial crisis, the significance of these stocks and indices as an investment vehicle grew. The IFM, according to Ejaz and Khan (2014), showed resilience during the GFC, which they attribute to a built-in risk-sharing element in Islamic securities contract design.

The COVID-19 pandemic presents other shocks to financial markets globally (Hung and Vo, 2021). For instance, as a consequence of the panic, a phenomenon induced by COVID-19 fear emerged in several markets, resulting in a scarcity of food (Agyei et al., 2021) and daily items in supermarkets, as well as a decrease in stock prices. As Owusu Junior et al. (2021) submit, on 16 March 2020, the stock market in the United States fell by 12% due to COVID-19 concerns, with all 11 groups in the S&P500 dropping. Share prices in Asia and Europe dropped as well, while bond yields fell in most areas of Europe, where a gauge of market stress reached levels not seen since the EDC of 2011/12. Following a decrease in daily new cases, most equities rose on 6 April 2020. COVID-19 has been shown to be contagious when it comes to financial assets (Fassas, 2020). This data backs up the ideas of the efficient market hypothesis (EMH), as it is called among its proponents. The EMH is premised that most stock market prices are appropriately valued based on the available information (Fama, 1970, 1998). In an efficient market, all accessible pertinent information about a financial asset is used in determining current prices to reflect the fact that the ideal projected return is equal to the market equilibrium return. Inferred future economic activity knowledge is a significant conditioning element that influences present financial asset prices.

Therefore, we argue that general uncertainties – primarily caused by the COVID-19 outbreak – are likely to elicit a response from global financial markets. Indeed, the COVID-19 pandemic has proved to be infectious when it comes to financial assets and scholars (see, e.g., Bossman, 2021; Bossman et al., 2022; Hassan et al., 2020; Hassan et al., 2020; Owusu Junior et al., 2021; Suleman et al., 2021; Yarovaya et al., 2021; etc.) have made contributions to explain the effects of the pandemic on asset classes. However, it is still unclear if Islamic stocks offer investors a safety net or insurance during a crisis. Given the conclusion of Lee and Goh (2016) that conventional financial markets are much integrated, which lessens opportunities for portfolio diversification, there is the need to examine the interrelations and connectedness of conventional and alternative asset classes amid novel episodes of financial crises (Bossman, 2021; Bossman et al., 2022).

Empirically, it is shown that Shariah-compliant stocks, which emanate largely from Islamic markets, are gaining considerable proportions in international portfolios for diversification, hedging, and safe haven benefits (Bossman, 2021; Bossman et al., 2022; Ng et al., 2020). The fundamental reason is the extent of integration among conventional markets which gradually washes away investors’ preference for them. Furthermore, Islamic stocks are proven to outperform their conventional equivalents during financial crises (Hassan et al., 2020; Shahzad et al., 2018). Notwithstanding, a new trading phase is occasioned by the COVID-19 pandemic (Hung and Vo, 2021) such that with previous crises being caused primarily by intrinsic factors, the tumult trading phase aroused by the COVID-19 are exogenous to the pandemic (Agyei et al., 2022, Quinsee, 2021). Therefore, for the sake of portfolio management vis-à-vis Islamic and conventional assets, the questions to be answered include, but are not limited to, the following: *(i)* do we expect the fundamental relationship between Islamic and conventional stocks to remain the same in the COVID-19 era?; *(ii)* to what extent are stocks from Islamic and conventional markets connected in stress periods?; *(iii)* does the connectedness between Islamic and conventional stocks differ across investment horizons?; *(ii)* does the connectedness between Islamic and conventional markets evolve from interdependence or contagion?; *(iv)* which markets transmit or receive the most shocks among Islamic and conventional markets?

Despite the presence of existing studies on Islamic and conventional markets (Bossman et al., 2022; Hassan et al., 2020; Shahzad et al., 2018; Yarovaya et al., 2021), the chance to investigate the problem further is provided by the volatility spillover index, which is especially important for portfolio investors. With the volatility spillover index, we can determine the direction(s) of volatilities among Islamic and conventional stocks; we are also able to assess the dynamic connectedness between stock markets (Salisu et al., 2020). Knowing the direction of spillovers in the time-frequency domain is essential to asset allocation and international portfolio management. For all investor classes, such as portfolio managers, speculators, and institutional investors, the total and pairwise dynamic interrelations provided by the spillover indices would facilitate asset allocations across diverse investment horizons. The opportunity for determining high and low asset connectedness periods across timescales is offered by the spillover indices, which is essential at this time of the COVID-19 pandemic owing to the heterogeneous and adaptive market behaviour of market participants (Asafo-Adjei, Owusu junior, & Adam, 2021; Bossman, 2021; Bossman et al., 2022; Ijasan et al., 2021; Owusu junior et al., 2021).

With the intensified growth of Islamic financial markets, arousing the interest of individual and institutional investors globally in including Islamic assets in portfolios, we maintain that this study is timely. To contribute to the growing literature on the COVID-19 pandemic and resilience of the Islamic markets, we conduct a comparative analysis of volatility spillovers between Islamic and conventional markets to examine the dynamism and asymmetries in the connectedness of these markets by applying the Baruník and Křehlík (2018) spillover methodology.

Our contribution to the literature on volatility spillover in the context of Islamic finance is manyfold. First, our study addresses the drawback of analysing aggregate volatility spillovers across markets, which may obscure valuable information for fund allocation and risk management. In examining volatility spillovers and the connectedness between stocks in Islamic and conventional markets in the short-, medium-, and long-term periods, we take into account investor heterogeneity in terms of investment choice and risk preference.

Second, market players’ emotions, expectations, and risk preferences vary and change over time. Speculators and hedgers are interested in short-term investments, while institutional investors and market regulators are interested in medium-term investments. As a result, while making investment choices and executing long-term plans, the time-investment element is critical. To do so, we look at how the complex connections between the various Islamic and conventional stock markets have evolved through time and at different (i.e., high, medium, and low) frequencies. Consequently, time-frequency analysis is appropriate to cater for the adaptive, heterogeneous, and complex behaviour of market participants. Nonetheless, the response offered by market participants to market shocks results in differing connectedness between markets over time (Bossman, 2021; Bossman et al., 2022; Owusu Junior et al., 2021). Thus, various investment horizons need to be considered when assessing spillovers between financial markets. This makes time-frequency analysis appropriate and, hence, its application in our study.

Third, we use the BK-18 methodology which is a build-up of the DY-12 spillover index. The DY-12 spillover index rather implies that investors behave similarly in markets and that spillover is unaffected by investment horizons, implying that it is the same in the short-, medium-, and long-term. To get around this restriction, we use the BK-18 spillover index, which is based on heterogeneous shock frequency responses. The BK-18 index offers valuable information on the intensities and directions of spillovers in the time-frequency domain, which is critical for determining the source and magnitude of contagions, and the market receiver of shocks. It also simultaneously investigates the volatility connectivity across markets over time and across different frequencies. By isolating the frequency domain spillover effects from the aggregate risk spillover effects, this decomposition provides a substantial benefit to market players. Investors may optimise their financing allocation and hedge their position against severe falling prices by distinguishing the frequencies. The notion that markets players work on distinct investment horizons is primarily motivated by the development of investor preferences (Agyei et al., 2022).

Furthermore, rather than employing aggregated indices for the conventional and Islamic markets, we conduct our analysis on country-specific markets to reveal the different dynamics that may prevail in each market and pair of markets. This would offer a broader picture to investors to undertake optimal investment decisions.

We find little evidence of any sporadic volatilities for Islamic stocks during the COVID-19 period across all frequencies relative to G7 stocks which showed some traces of clusters during the COVID-19 period studied, suggesting the relative resilience of the Islamic stocks over their conventional counterparts, specifically, G7 stocks. More significantly, we infer contagion occurrences evidenced by increased spillovers in 2017/18 and 2020/21, which are due to Brexit and the COVID-19 pandemic respectively. Additionally, we explicate that spillovers between Islamic and G7 markets are largely contributed by short-term dynamics and, hence, institutional investors stand a chance to benefit from Islamic stocks during market shocks. Speculators and hedgers may focus on Islamic assets only in the medium-to long-term when G7 stocks are contained in their portfolios.

The remainder of the paper is organised as follows. We review related literature in Section 2; Section 3 details our methodology; data and preliminary results are presented in Section 4; empirical results are discussed in Section 5. We provide practical implications in Section 6 and conclude in Section 7.

## 2 Literature review

Investor behaviour tends to change over time, especially during difficult periods like the ones presented by the COVID-19 pandemic. Because markets do not operate in a vacuum, asymmetric and time-based investor behaviour is reflected in market pricing. The adaptive markets hypothesis (AMH) of Lo (2004) and the heterogeneous markets hypothesis (HMH) of Müller et al. (1993) are two hypotheses that support this occurrence. The HMH hypothesises that various economic agents make investment decisions across different time horizons based on their risk and return preferences by analysing historical and current news. Ideally, we could redefine time as intrinsic time, which relates to time scales of short-, medium-, and long-term, to account for time horizon. Through the HMH, investors are led to switch to or include several asset classes in their portfolios during market stress for hedging and diversifying risks.

The AMH and HMH are summed up by Owusu Junior et al. (2021) to coin the competitive markets hypothesis (CMH). The CMH posits that during crises, spillovers and information flow between assets and/or asset classes intensify owing partly to the relentless search by rational, yet irrational market participants for competitive risks and returns to satisfy portfolio objectives, i.e., minimising risk whilst maximising returns. Naturally, market participants' expectation of the financial markets’ responsiveness to intensified spillovers and information in uncertain periods like the one occasioned by the COVID-19 pandemic would result in rowdy trading of assets, causing unexpected non-fundamental connectedness between assets and/or asset classes (Bossman, 2021; Bossman et al., 2022). This has influenced the focus of recent empirical works vis-à-vis financial markets.

A slew of research has reviewed the fundamental concept of portfolio diversification in pursuit of competitive returns and risk levels as a result of previous financial crises and the present COVID-19 pandemic. The notion that investors are constantly searching for conflicting risks and rewards, and that this search increases under stressful market circumstances, runs across several studies (Adam, 2020; Agyei et al., 2021; Asafo-Adjei et al., 2020; Asafo-Adjei, Adam and Darkwa, 2021; Baur and Lucey, 2010; Chkili et al., 2021; Bossman, 2021; Bossman et al., 2022; Hung and Vo, 2021; Mensi et al., 2020; Owusu Junior et al., 2021; Owusu Junior, Tiwari, Padhan and Alagidede, 2020; Owusu Junior, Adam and Tweneboah, 2020; Owusu Junior and Tweneboah, 2020; etc.).

Due to its size, continued growth, and stable performance during and after recent financial crises, risk diversification via exposure to Islamic equity markets has become more appealing to investors (Balli et al., 2019; Hassan et al., 2020). Greater portfolio diversity requires in-depth knowledge of the co-movements, interdependencies, and spillovers among the asset classes and markets under consideration. The majority of relevant research is limited to either developed markets or the use of aggregated (composite) Islamic indices. The market-specific dynamics, especially for Islamic markets, are yet to be fully revealed by the literature.

The DJ World Islamic (DJWI) and DJ World Islamic Financial (DJWIF) indexes, as well as Islamic equity indices from Japan, the United States, and the United Kingdom, are modelled for negative and positive spillover effects, systemic and tail-dependent risks by Shahzad et al. (2018) over the period 01 January 1996 to 31 December 31 2015. Their methodological approach included a Value-at-Risk (VaR), conditional VaR (CoVaR), Delta conditional VaR (ΔCoVaR), canonical vine conditional VaR (c-vine CoVaR), vine copula, and static and time-varying bivariate techniques. They document significant changes in market spillovers during the studied crisis period. Balli et al. (2019) examine the total, net, and pairwise return and volatility spillovers across 15 Islamic equities markets with data between 2007 and 2017. The authors find rising interactions in return and volatility spillovers using the generalised VAR-based spillovers index. They divulge that the magnitude of spillovers is asymmetric between Islamic markets and in times of crisis, aggregate spillovers across Islamic equities markets become more intense.

Hassan et al. (2020) utilise the threshold generalised autoregressive conditional heteroscedasticity (TGARCH) and generalised forecast error variance decomposition (GFEVD) to calculate time- and frequency-domain volatility spillover for Islamic and conventional stocks as well as crude oil in the BRICS nations, providing investors with information on the amount and speed of the volatility spillover. Their findings reveal that the overall volatility spillover is mostly driven by a long-term component and as a result, recommend that investors with short- and medium-term investment goals might consider these assets. Ng et al. (2020) extend the heterogeneous autoregressive (HAR) with GARCH, asymmetric effects, and jump-robust volatility estimator established in a multivariate setting to investigate the realised volatility transmission between the Malaysian Islamic market and various global sectoral Islamic stock markets using the nearest neighbour truncation approach. The results, which were based on intraday data, indicate that Islamic equities' daily realised volatilities are heavily influenced by their ‘own’ short-, mid-and long-term volatility components.

Haddad et al. (2020) use Centoni, Cubadda and Hecq's (2007) permanent-transitory (P-T) decompositions to study the importance of permanent versus transitory shocks, as well as their domestic and foreign components, in explaining the business cycle fluctuations of seven Dow Jones Islamic stock markets (DJIM), namely the US, UK, Canada, Europe, Asia-Pacific, Japan, and GCC, from April 2003 to November 2018. Additionally, they employ the Diebold and Yilmaz (2012) (DY-12) estimator to examine how these shocks spread across Islamic stock markets and a set of global risk variables. The findings of the P-T decomposition indicate that the DJIM U.S., U.K., Europe, and GCC indices are sensitive to both domestic and international shocks, whereas the DJIM Canada, Japan, and Asia-Pacific are more susceptible to domestic shocks.

Through the DY-12 approach, Haddad et al. (2020) reveal that during the financial upheaval, the degree of return and volatility spillover increases, indicating that the contagion phenomenon is at work; return and volatility spillovers are mostly transmitted by the DJIM US, whereas return and volatility spillovers are primarily received by the DJIM GCC; the Dow Jones Islamic stock indices are only sporadically connected to global risk concerns. Yarovaya et al. (2021) investigate the influence of the COVID-19 pandemic on stock and bond market spillovers across conventional and Islamic markets and produce findings suggesting that Islamic bonds (Sukuk) provide safe haven opportunities during the COVID-19 pandemic, whereas spillovers between conventional and Islamic stock markets become larger throughout the pandemic.

Mensi et al. (2021) investigate the frequency of crude oil futures spillovers to the Middle East and North Africa (MENA) stock markets using the DY-12 and Baruník and Křehlík (2018) (BK-18) methods, in addition to the wavelet methodology. The authors reveal time-varying volatility spillovers, indicating that short-term spillovers are more significant than intermediate-term spillovers. Mensi et al. (2021) present that the major contributors of spillovers in the short and intermediate periods are Saudi Arabia, Qatar, and the United Arab Emirates (UAE). In the short run, Brent oil, Egypt, Morocco, and Turkey are net recipients of spillovers, but in the intermediate term, they become net transmitters. In Mirz, Rizvi, Saba, Naqvi and Yarovaya's (2021) analysis of the risk-adjusted performance of Islamic and conventional stock funds during the COVID-19 pandemic, Islamic equities outperformed their conventional equivalents in terms of risk-adjusted performance, investing strategies, and volatility timing. The findings showed that Islamic equities are more robust to COVID-19 shocks than non-Islamic counterparts during the pandemic's peak months, outperforming non-Islamic markets.

The existing works on Islamic and conventional markets have failed to infer or employ methods that reveal contagion,^1^ and its source(s) and magnitude. Whiles Balli et al.’s (2019) study does not extend to the prevailing COVID-19 pandemic era, the works of Mensi et al. (2021) and Mirz et al. (2021) do not capture contagion that may be present to the individual Islamic indices. The question of whether a spillover is an interdependence or contagion (Forbes and Rigobon, 2002) is still being debated in the literature (see, e.g., Owusu Junior, 2020; Owusu Junior, Alagidede and Tweneboah, 2020; etc.). Besides, the COVID-19 pandemic has been credited with some shocks to the global economy (Adam, 2020; Agyei et al., 2021; Bossman, 2021; Bossman et al., 2022; Owusu Junior et al., 2021). Therefore, studies that examine the volatility spillovers across and among asset classes need to incorporate contagion and assess its magnitude and sources.

As Quinsee (2021) documents, the shocks to financial markets in the era of the COVID-19 pandemic is exogeneous to the pandemic. The persistence of these shocks in the COVID-19 era warrants that empirical works need to evaluate the presence of contagious spillovers, their magnitude and sources. Our review of the extant literature reveals that attention to this phenomenon is lacking in the context of individual Islamic and conventional stock markets. A contribution towards this direction is thus essential during the COVID-19 pandemic. Consequently, a vibrant strand of the ever-growing empirical literature on the effects of the pandemic in financial contagion emerges.

Based on a Bayesian time-varying parameter vector autoregressive technique, Fassas (2020) explores the dynamic connectivity across the variance risk premium in international advanced and emerging equities markets. Fassas reports a significant, albeit diminishing, level of interconnectivity across investor sentiment in the US, developed, and emerging markets under consideration until early 2020. However, following the COVID-19 pandemic, overall investor risk aversion connectedness improves, but its dynamics change, demonstrating that emerging market risk aversion is a significant contribution to international markets connectedness. The significant change in overall investor risk aversion connectedness suggests financial contagion. Using realised volatility data from sixteen major stock markets globally, Liu et al. (2021) investigate risk contagion among international stock markets during the COVID-19 pandemic. Based on the DY-12 and BK-18 connectedness approaches, the authors report that the COVID-19 outbreak considerably amplifies the risk contagion effects in international stock markets. They also report that risk spillovers from stock markets in Europe and the United States are fast increasing, whilst risk spillovers from Asian markets are decreasing following the start of the COVID-19 pandemic.

Using the DY-12 spillover index and wavelet coherence, Hung and Vo (2021) examine the time-frequency connectedness and spillover effects between the S&P 500, crude oil prices, and gold assets. They assess whether the time-varying dynamic return spillover index reflected the intensity and direction of transmission during the COVID-19 outbreak. The authors report that return transmissions are more visible during the COVID-19 crisis. Akhtaruzzaman, Boubaker and Sensoy (2021) examine how financial contagion occurs between China and G7 nations through financial and non-financial enterprises. Their empirical findings reveal that listed companies in these nations, both financial and non-financial, have much higher conditional correlations between their stock returns. However, during the COVID-19 pandemic, the size of the rise in these correlations is significantly larger for financial businesses, suggesting the importance of their participation in financial contagion transmission.

The influence of the COVID-19 outbreak on the time-varying connection between stock and bond returns is investigated by Papadamou et al. (2021) using both a panel data specification and wavelet analysis. The authors uncover flight-to-quality episodes during the COVID-19 worldwide pandemic crisis using daily data on bond and stock returns for 10 nations throughout Europe, Asia, the United States, and Australia. Additionally, the authors underscore that flights take place concurrently in several countries and are not country-specific phenomena, which corroborates the principles of financial contagion.

We notice that the literature on financial contagion is limited between Islamic and conventional markets despite the growing interest of market participants in Islamic assets for asset allocation portfolio diversification in recent periods (Bossman, 2021; Bossman et al., 2022; Ng et al., 2020). This ignites our motivation to study the connectedness between Islamic and conventional markets covering the COVID-19 pandemic era.

### 2.1 Motivation

Although information moves across markets as a result of investors' searches, spillovers and information flow intensify during times of market stress. This situation is an epitome of Owusu Junior et al.’s (2021) competitive market hypothesis (CMH), which implies that the intensity of information flows and spillover between markets of the same and different asset classes is aggravated in part by rational, though somewhat irrational investors' relentless search for competing rewards and risks to meet portfolio goals.

Some scholars have made initial contributions towards the interrelationships between Islamic and conventional markets (Balli et al., 2019; Bossman, 2021; Bossman et al., 2022; Haddad et al., 2020; Hassan et al., 2020; Mirz et al., 2021; Ng et al., 2020; Shahzad et al., 2018; Yarovaya et al., 2021, etc.). These initial studies, though make significant contributions to the literature, no such study has yet examined the extent, magnitude, and direction of spillovers between Islamic and conventional stock markets using the spillover index approach whilst incorporating the adaptive and heterogeneous behaviour of market participants.

Following the principles of the CMH, Bossman (2021) and Bossman et al. (2022), for instance, examine the connectedness between Islamic and conventional markets using transfer entropy techniques. Balli et al.’s (2019) study does not extend to the COVID-19 period and is also focused solely on Islamic markets. In uncertain times like the COVID-19 era, international investors would be interested in combining faith-based assets with conventional ones for portfolio diversification benefits and, hence, a comparative analysis is essential at this time of the pandemic. Other works (Hassan et al., 2020; Mirz et al., 2021; Ng et al., 2020; Shahzad et al., 2018; Yarovaya et al., 2021), although focus on the connectedness of Islamic and conventional markets, their contributions are insufficient to reveal the magnitude, direction, and sources of spillovers between the two broad markets, which serve as distinct asset classes. Also, no such study assesses contagion between Islamic and conventional markets in the COVID-19 era.

To fully complement the principles of the CMH and assess its operability in the uncertain times of the COVID-19 pandemic, we add to the growing strand of empirical literature in the COVID-19 era by employing the dynamic spillover connectedness approach to examine the connectedness between Islamic and conventional stock markets. Specifically, we employ the spillover index method proposed by Baruník and Křehlík (2018) to examine the dynamic connectedness between selected Islamic and G7 stock markets. This method aids in ascertaining the size, direction, and sources of spillovers between Islamic and conventional stocks. In the spirit of the AMH and HMH, we conduct our analysis in both time and frequency domains using rolling windows that result in frequency bands. More importantly, as a supplementary analysis, we employ the TVP-VAR connectedness approach to confirm the robustness of our findings.

## 3 Methods

We employ the Baruník and Křehlík (2018) (BK-18) spillover index to examine the dynamic connectedness and spillovers between Islamic and conventional stock markets to reveal the time- and frequency-domain dynamics of the two asset classes during different market conditions.

### 3.1 The BK-18 spillover index

Baruník and Křehlík (2018) use generalised forecast error variance decompositions (GFEVDs) to quantify connectivity, as inspired by Diebold and Yilmaz (2012). The matrix of a vector autoregressive (VAR) model with local covariance stationarity is used to decompose the data. We represent a K-variate procedure, $Y_{t}={\left(y_{1,t},\ldots ,y_{K,t}\right)}^{\prime }$ given t=1,…,T and a VAR(ρ) which may be expressed as

(1) $$Y_{t}=\overset{p}{\underset{i=1}{\sum }}\varphi_{i}y_{t-i}+\varepsilon_{t,}$$

where coefficient matrices and white noise with (prospective non-diagonal) covariance matrix Π are denoted as $\varphi_{i}$ and $\varepsilon_{i}$. A regression is carried out between each variable in the system (1) and its ‘own’ ρ lags and the ρ lags of all the remaining variables. Accordingly, φ holds wide-ranging information on the relationships between all variables. The expediency of working with a (K×K) matrix $\left(I_{K}-\emptyset_{1}L-\ldots -\emptyset_{p}L^{p}\right)$ with identity $I_{K}$ must be moted. The VAR system is characterised by a moving average MA(∞) when the roots of the representative equation |θ(z)| lie outside of the unit circle

(2) $$Y_{t}=\psi \left(L\right)\varepsilon_{t},$$

with ψ(L) depicting an infinitely lagged polynomial. The role of the kth variable, known as the GFEVD, to the variance of forecast error of the element j can be written as

(3) $${\left({\text{Θ}}_{H}\right)}_{j,k}=\frac{\sigma_{kk}^{-1}\sum_{h=0}^{H}\psi_{h}\text{Π}){\left(\psi_{h}\text{Π}){\left(\psi_{h}\text{Π}\right)}_{j,k}\right)}^{2}}{\sum_{h=0}^{H}{\left(\psi_{h}{\text{Π}}_{h^{\prime }}\right)}_{j,k}},$$

where h=1,…,H and $\sigma_{kk}=\left({\text{Π}}_{kk}\right)$. This could hold since the measure of connectedness is contingent on decomposed variance, which are the transformations of $\psi_{h}$ and serve as the contribution of the shocks to the system. Because row contributions do not aggregate to 1, for the sake of completeness, a standardisation of the matrix ${\text{Θ}}_{H}$ is generated as

(4) $${\left({\tilde{\text{Θ}}}_{H}\right)}_{j,k}=\frac{{\left({\text{Θ}}_{H}\right)}_{j,k}}{\sum_{k=1}^{N}{\left({\text{Θ}}_{H}\right)}_{j,k}}.$$

The pairwise connectivity (Eq. (4)) may be aggregated for overall connectedness in a system. In line with Diebold and Yilmaz (2012), this may be defined as the proportion of variation in predictions provided by errors other than own error (which is the same as the ratio of the off-diagonal components' sum to the whole matrix's sum.) as shown in

(5) $$C_{H}=100*\frac{\sum_{j\neq k}{\left({\tilde{\text{Θ}}}_{H}\right)}_{j,k}}{\sum {\tilde{\text{Θ}}}_{H}}=100*\left(1-\frac{Tr\left\{{\tilde{\text{Θ}}}_{H}\right\}}{\sum {\tilde{\text{Θ}}}_{H}}\right),$$

where Tr{.} represents the operator for tracing, and the arithmetic aggregate of all elements in the matrix is the denominator. As a result, connectedness denotes the forecast variance's relative contribution to the system's other variables. As a result, bi-directional connectivity may be assessed (*“to”* and/or *“from”* market i from all other markets k). The difference between *“to”* and *“from”* spillovers is also used to calculate *“net”* connectivity. As a result, a market with a positive net spillover acts as a “net transmitter,” while one with a negative spillover acts as a “net receiver” of shocks.

The spectral representation of connectivity is shown at this point. With a frequency response function of $\psi {\left(e\right)}^{-i\omega }=\underset{h}{\sum }e^{-i\omega h}\psi_{h}$ of coefficients that could be transformed by Fourier transforms $\psi_{h}$ with $i=\sqrt{-1}$, a spectral density of $Y_{t}$ at frequency, ω can be defined as MA(∞) filtered series

(6) $$S_{y\left(\omega \right)}=\overset{\infty }{\underset{h=-\infty }{\sum }}E\left(Y^{\prime }Y_{t-h}\right)e^{-i\omega h}=\psi \left(e^{-i\omega }\right)\text{Π}\psi^{\prime }\left(e^{+i\omega }\right).$$

where $S_{y\left(\omega \right)}$ is the power spectrum which details the distribution of the variance of $Y_{t}$ over the frequency components ω. The causation spectrum over ω∈(−π,π) is defined in (7); noting that it reflects the fraction of the ith variable attributable to shocks in the kth variable at a particular frequency ω. As a consequence,

(7) $${\left(F\left(\omega \right)\right)}_{j,k}=\frac{\sigma_{kk}^{-1}|\psi \left(e^{-i\omega }\right){\text{Π}}_{j,k}{|}^{2}}{{\left(\psi \left(e^{-i\omega }\right)\text{Π}\psi^{\prime }\left(e^{+i\omega }\right)\right)}_{j,j}}$$

could be understood as *within-frequency* causation due to the denominator. To get a natural decomposition of GFEVD to frequencies, we weigh ${\left(F\left(\omega \right)\right)}_{j,k}$ by the frequency share of the variance of the jth variable. We define the weighting function as

(8) $${\text{Γ}}_{j}=\frac{{\left(\psi \left(e^{-i\omega }\right)\text{Π}\psi^{\prime }\left(e^{+i\omega }\right)\right)}_{j,j}}{\frac{1}{2\pi }\int_{-\pi }^{\pi }{\left(\psi \left(e^{-i\lambda }\right)\text{Π}\psi^{\prime }\left(e^{+i\lambda }\right)\right)}_{j,j}d\lambda }$$

summating to real-valued^2^ numbers up to 2π and represents the index of the jth variable at a particular frequency. Connectivity must be measured across periods in practical financial applications. As a result, rather than measuring connectedness at single frequencies, it is more appropriate to do so across frequency bands. We take a formal representation of frequency band, d, as d=(a,b):a,b∈(−π,π),a<b, for which we define the GFEVDs as

(9) $${\left({\text{Θ}}_{d}\right)}_{j,k}=\frac{1}{2\pi }\overset{b}{\underset{a}{\int }}{\text{Γ}}_{j}\left(\omega \right){\left(F\left(\omega \right)\right)}_{j,k}d\omega .$$

A scaled^3^ generalised variance decomposition may be constructed in the same frequency band d as

(10) $${\left({\tilde{\text{Θ}}}_{d}\right)}_{j,k}={\left({\text{Θ}}_{d}\right)}_{j,k}/\underset{k}{\sum }{\left({\text{Θ}}_{\infty }\right)}_{j,k}.$$

Then, the *within-frequency* and frequency connectivity across d are expressed in (11(11) and (12)(12), respectively.

(11) $$C_{d}^{W}=100.\left(1-\frac{Tr\left\{{\tilde{\text{Θ}}}_{d}\right\}}{\sum {\tilde{\text{Θ}}}_{d}}\right)$$

(12) $$C_{d}^{F}=100.\left(\frac{\sum {\tilde{\text{Θ}}}_{d}}{\sum {\tilde{\text{Θ}}}_{\infty }}-\frac{Tr\left\{{\tilde{\text{Θ}}}_{d}\right\}}{\sum {\tilde{\text{Θ}}}_{\infty }}\right)=C_{d}^{W}.\left(\frac{\sum {\tilde{\text{Θ}}}_{d}}{\sum {\tilde{\text{Θ}}}_{\infty }}\right)$$

It is important to note that $C_{d}^{W}$ represents the connectivity that occurs inside a frequency band and is only weighted by the series’ power on that frequency band. $C_{d}^{F}$, on the other hand, breaks down overall connectivity into discrete pieces that add up to the original connectedness metric, as presented by Baruník and Křehlík (2018). (π+0.00001,π/4,π/16,π/32,π/64,0) are the frequency bands we utilise, which is in line with the extant literature (Baruník and Křehlík, 2018; Tiwari et al., 2018; Tiwari et al., 2019; Owusu Junior, Alagidede and Tweneboah, 2020). Table 1 shows the daily ranges that correspond to the relevant bands.

**Table 1:** Interpretations to frequency bands.

Frequency	Bands	Days	Interpretation
$d_{1}$	3.14–0.79	1–4	Intraweek
$d_{2}$	0.79–0.20	4–16	Week-to-fortnight
$d_{3}$	0.20–0.10	16–32	Fortnight-to-month
$d_{4}$	0.10–0.05	32–64	Month-to-quarter
$d_{5}$	0.05–0.00	64∼∞	Quarter-and-beyond

## 4 Data and preliminary results

The daily stock market indices for 17 key Islamic markets (Bahrain, Bangladesh, India, Malaysia, Indonesia, Kazastan, Pakistan, Egypt, Iraq, Jordan, Kuwait, Oman, Palestine, Qatar, Saudi Arabia, United Arab Emirates (UAE), and Morocco)^4^ and G7 economies (Canada, France, Germany, Italy, Japan, UK, and the USA)^5^ are utilised in the processing and analysis. To concentrate on country-specific stock markets that make up the Islamic and conventional markets, we select the stock market indices for countries that have Islamic stock indices. The choice of Islamic markets was influenced by the availability of data and our sample is similar to that of Balli et al.’s (2019) who employ 15 Islamic indices to examine the spillover determinants within Islamic markets between 2007 and 2017. Their study covers Islamic markets only whilst the period does not extend to the COVID-19 pandemic. We proxy conventional stock markets with G7 markets. These markets form a group of seven advanced economies with significant contributions to the global financial market.

The dataset spanned between 23 November 2015 and 08 September 2021, yielding 662 common data observations. The daily stock indices were supplied by *EquityRT* and are expressed in USD. The log-returns of the daily stock indices were computed as

(13) $$r_{t}=lnP_{t}-lnP_{t-1},$$

where $r_{t}$ defines the continuously compounded returns, $P_{t}$ represents the price of an asset in period t, and $P_{t-1}$ represents the price of an asset in the previous period t−1.

A forecast horizon (H) of 100 days is utilised, as well as a 100-day rolling window. This aggregate to a little over a quarter of a year, and it is sufficient to accommodate for time differences. The rolling window framework eliminates the need for crisis start and end dates to be specified exogenously. By displaying the resultant spillover indices, we can account for significant changes in the form of spillovers throughout the sample period, as advocated by Yilmaz (2010) and Owusu Junior et al., 2020a, Owusu Junior et al., 2020b, Owusu Junior et al., 2020c.

A trajectory of the stock indices for all the countries is presented in Figure 1. The Shapiro-Wilk test of normalcy confirms skewness and excess kurtosis (see Table 2). The resulting statistics for skewness and kurtosis respectively depict non-normal and leptokurtic distributions across the studied markets. Asymmetries in return distributions are confirmed by these findings. This offers a strong incentive to use the BK-18 approach – relative to the DY-12 time-invariant approach – to examine the dynamic and asymmetric connection between Islamic and conventional stocks. Traces of volatilities may also be seen in the time series returns plots in Figure 2, indicating that the series is generating time-varying risk. The mean returns (see Table 2) on stocks over the entire sample were positive for all countries except for Egypt, Iraq, and Oman which recorded negative mean returns over the studied period.

**Figure 1:** Time series plot of Islamic and G7 stock indices.

**Table 2:** Descriptive summary of the studied Islamic and G7 stock markets.

Panel A	Bahrain	Bangladesh	Egypt	India	Indonesia	Iraq	Jordan	Kazastan	Kuwait	Malaysia	Morocco	Oman
Observations	662	662	662	662	662	662	662	662	662	662	662	662
Mean	0.0005	0.0003	-0.0004	0.001	0.0001	-0.0006	0	0.0012	0.0008	0	0.0005	-0.0005
Std. Dev	0.0086	0.0126	0.026	0.0162	0.0186	0.0157	0.0071	0.0148	0.0146	0.0134	0.0113	0.008
Skewness	-3.3389	0.1637	-6.3596	-1.1697	-1.7245	-3.6806	-0.6125	-0.1226	-3.4147	1.0903	-5.2228	-1.0124
Kurtosis	36.5613	22.4701	91.3578	10.9623	13.1517	51.597	26.0454	10.1243	77.1436	51.4477	83.8503	12.4634
Normtest.W	0.7246	0.8024	0.6322	0.889	0.8625	0.7206	0.8039	0.877	0.5845	0.7289	0.7214	0.8685
**Panel B**	**Pakistan**	**Palestine**	**Qatar**	**Saudi**	**UAE**	**Canada**	**France**	**Germany**	**Italy**	**Japan**	**UK**	**USA**
Observations	662	662	662	662	662	662	662	662	662	662	662	662
Mean	0.0004	0	0.0004	0.0009	0.0007	0.0005	0.0009	0.0006	0.0007	0.0006	0.0007	0.0007
Std. Dev	0.0174	0.0066	0.0136	0.0168	0.0151	0.01	0.0114	0.0115	0.0127	0.0109	0.0108	0.0102
Skewness	-0.2314	-1.4588	-0.3555	0.969	-0.0644	-2.1785	0.0297	-0.3807	-0.3045	0.2011	-0.2519	-3.2868
Kurtosis	5.8883	28.3733	5.9793	37.6578	62.7044	22.9166	5.2053	3.5182	2.5067	3.8576	6.4973	38.9618
Normtest.W	0.9132	0.7711	0.9182	0.7536	0.6769	0.8674	0.9426	0.9529	0.9669	0.9608	0.9143	0.7897

**Figure 2:** Return series for Islamic and G7 stocks.

## 5 Empirical results

### 5.1 Time-frequency-domain analysis

The time-frequency-domain analysis under the BK-18 spillover index helps to establish whether or not there is contagion by accounting for the evolution of total connectedness over time. We advance our analysis by investigating the spillover effects between the Islamic and G7 stock markets at various frequencies. This decomposition attempts to account for market participants’ diverse expectations and desires across different time horizons. The short-, medium- and intermediate-term spillovers, classified into five frequency bands (intraweek, week to a fortnight, a fortnight to a month, month to quarter, and quarter and beyond) are reported in Table 3 for Islamic and G7 markets. The total and pairwise spillover tables for the isolated Islamic and G7 markets are supplied in the Appendix (Tables S1–S5). Pairwise plots are shown in Figures S1–S5 in the Appendix.

**Table 3:** Total and Net spillover indices across frequency bands for Islamic and G7 stocks.

Note: ^[a]^ “Absolute to” measures return spillovers from market/country j to other markets. “Absolute from” measures return spillovers from other markets to market j. ^[b]^Within to measures return spillovers from market j to other markets, including from own innovations to country k. Within from measures return spillovers from other markets to market j, including from own innovations to market k (see Owusu Junior et al., 2020a, Owusu Junior et al., 2020b, Owusu Junior et al., 2020c; Tiwari et al., 2018, 2019). The largest contributions of markets per frequency band are in bold italics. A positive ‘Net’ suggests that the country/market is a net transmitter while a negative ‘Net’ denoted net recipient market/country.

We observe from the net spillover indices for all the markets (Islamic and conventional) in Table 3 that spillovers in the very short-term (intraweek) are comparatively higher than in the medium-to long-term horizons. For instance, the return spillover within the first band, 3.14 to 0.79, which approximates to 1–4 days, is 40.13. This return spillover reduces to 15.04, 3.49, 1.75, and 0.88 respectively for the second (0.79–0.20), third (0.20–0.10), fourth (0.10–0.05), and fifth (0.05–0.00) bands. Similarly, the spillover is seen to be decreasing over time among both Islamic stocks only and among G7 stocks only. This finding is indicative that all the markets respond quickly to shocks in the first few trading days. At best, within the intraweek band over the period studied, the Islamic and conventional markets studied are more responsive to market shocks than in later days.

These results are consistent with Mensi et al.’s (2021) observations and also corroborate the EMH such that, in the short-term, asset prices fully reflect all pertinent information (Fama, 1970, 1998), resulting in high market dynamics at high frequencies. Using a similar methodology, Mensi et al. (2021) generate results that indicate that short-term spillovers are more significant than intermediate-term spillovers for Islamic and conventional markets, specifically BRICS economies. However, these observations are converse to those of Hassan et al. (2020) who utilise TGARCH and GFEVD to calculate time- and frequency-domain volatility spillover for Islamic and conventional stocks but revealed that the overall volatility spillover is mostly driven by a long-term component and as a result, recommended that investors with short- and medium-term investment goals might consider these assets. The differences in results may be attributed to differences in the methodological approaches.

Our findings reveal that when the selected Islamic and G7 markets are studied together, the largest contributors of shocks to these markets are France, UAE, and Malaysia in the high-frequency bands (short-term), notably in the first spillover band. Throughout the remaining spillover bands, Canada, Kuwait, and Saudi Arabia are found to be the largest contributors of shocks to the selected Islamic and G7 stock markets. On the other hand, across all spillover bands, we find Iraq to be the smallest contributor to the shocks between the markets studied. This implies that the Iraqi market has fewer shocks to present to other conventional markets.

Next, we isolate the two broad markets to study the transmission of volatilities across and within the markets. We identified, from the Islamic markets alone, that UAE and Malaysia offer the greatest contribution to market return spillovers in the very short-term (i.e., within band 3.14 to 0.79) and this corroborates the results of Balli et al. (2019), who found, inter alia, UAE and Malaysia as characterised by persistent volatility clusters between Islamic equities. Consistently, Kuwait and Saudi Arabia remain the greatest contributors of market spillovers to the selected Islamic markets over bands 2 to 5 with Iraq being the least contributor of return spillovers among the Islamic markets. For the G7 markets, France and Germany were found to be the significant contributors of volatility spillover across the markets. Japan, on the other hand, was found to make a relatively ‘insignificant’ contribution to volatility spillover to the G7 markets. Comparatively, we reveal that the G7 stock markets possess substantial volatilities across all time horizons than the Islamic stock markets.

Studying the markets together in terms of receiving market volatilities, we report that Saudi Arabia receives high levels of volatility spillover in the short-term, specifically in the spillover band 3.14 to 0.79. Between bands 2 and 5, Bahrain is found to be the recipient of the largest volatility spillover among the studied Islamic and G7 stock markets. When the broad markets are studied in isolation, UAE suffers more volatility spillovers from other Islamic markets in the spillover band 3.14 to 0.79, but from bands 2 to 5, Bahrain is the greatest recipient of volatility spillovers. Within the G7 markets, Germany suffers the greatest volatility spillover in the very short-term (3.14–0.79) whereas, within bands 2 to 5, France receives the greatest volatility spillovers.

We present the time-frequency subtleties of the return volatility among Islamic and G7 stocks in Figure 3^6^. Panel A shows the time-frequency dynamics of the return volatility for Islamic and G7 stocks altogether whereas Panels B and C represent, respectively, the return volatility of Islamic stocks only and G7 stocks only.

**Figure 3:** Overall rolling spillovers across frequency bands.

From the plots, we notice that the volatility spillovers are dominated in the short term for all samples. We spot a similar trajectory of spillovers across the frequency bands with differing magnitudes. In Panel A (the all-stocks sample), we notice variations in the spillover but largely between 38% and 50% in the short-term, with a few upsurges above 75% within 2017/18 and 2020/21. Akhtaruzzaman et al. (2021), Fassas (2020), Haddad et al. (2020), Liu et al. (2021), Papadamou et al. (2021), all reveal possible upsurges in markets connectedness in the short term in stressed market periods.

A separate analysis of the two markets reveals that the G7 stocks are prone to high volatility spillovers relative to the Islamic stocks. Whereas the spillover across Islamic markets is relatively stable during the COVID-19 period (between 2020 and 2021), the spillovers are more observable in G7 stocks especially in the short-term across spillover bands 1 and 2 (intraweek and week-to-fortnight). This suggests that conventional stocks are susceptible to more volatilities than Islamic stocks. These findings are in line with the works of Balli et al. (2019), Liu et al. (2021), Mirz et al. (2021), Shahzad et al. (2018), etc. Besides finding support for our findings, the results shown in the plots (Figure 3) are consistent with those reported in the spillover tables (see Table 3 and the results in the Appendix). We find little evidence of any sporadic volatility for Islamic stocks during the COVID-19 period across all frequencies, particularly in the short term.

On two occasions (2017/2018 and 2020/2021), we discover, through inference, financial contagion across all spillover bands (see Figure 3). Notably, our results reveal the development of contagion within 2017 where we identify substantial increases in spillover connectedness between the studied Islamic and G7 markets, which corroborates the definition of contagion by Forbes and Rigobon (2001, 2002). At high frequencies (in the short-term), we observe surging volatilities (about 90%) for all markets and reduce across spillover bands 2 to 4. In line with Mensi et al. (2021), we could attribute this contagion to the slowdown in economic activities experienced by China in 2017 and/or the delayed effects of the substantial losses borne by global investors on 24 June 2016 following the referendum that confirmed Britain's exit (Brexit) from the European Union (David, 2016). Brexit caused investors in global stock markets to lose over US$2 trillion, making it the biggest single-day loss in history.

Given that the sudden increases in spillovers across the bands occurred in 2017/18, we infer the delayed contagion hypothesis as posited by Boako and Alagidede (2017). We attribute the spike in spillover connectedness in 2020/2021 to the turbulent market conditions introduced to financial markets by the COVID-19 pandemic. The traces of contagion are also spotted for the separate spillover plots for Islamic and G7 stocks as projected by Figure 3. It is essential to note that the sources of the inferred contagion are France, UAE, and Malaysia (in the short-term) and Canada, Kuwait, and Saudi Arabia (in the medium-to-long-term horizon), who happen to be the largest contributors or transmitters of shocks across all studied markets. With UAE and Malaysia's inclusion in the originators of contagion, Balli et al.’s (2019) results are corroborated.

We assess possible causes of the intensified spillovers during Brexit and the COVID-19 pandemic. for the Brexit, the exit of Britain from the European Union might have case a negative signal to international investors concerning their portfolio holdings. In responding to such a negative signal, all responses in the short term are attributable to transitory factors, which are likely to affect cross-market correlations (Jena et al., 2021), which then causes a significant change in the fundamental connectedness between markets. Owusu Junior et al. (2021), Bossman (2021), and Bossman et al. (2022) note that market dynamics and connectedness in the medium- (long-) term are attributable to key events (fundamental factors). Thus, in the short term, transitory factors emanating from panic decisions and herd behaviour result in extreme connectedness, as confirmed by our results. In the medium term, key events in the market also drive the connectedness between assets. Such connectedness may last throughout the specific event. We spot such connectedness in the Brexit case and that of the COVID-19 is not an exception. In the long-term, where markets are saturated with information flow within and across markets, spillovers and connectedness are attributable to the fundamental or longstanding relationships between markets (assets and/or asset classes).

In the COVID-19 era, the studied Islamic and conventional markets seem to respond to the negative information flow concerning the spread of the coronavirus (Bossman, 2021; Hung and Vo, 2021). The fears surrounding the pandemic could cause investors to make temporal decisions concerning their investment holdings. The pandemic is associated with health risks, which causes several uncertainties in areas such as income generation, etc. These uncertainties tend to affect business operations. More importantly, lockdowns or stay-at-home restrictions that were embarked upon by several countries worldwide caused severe impacts on business activities (Agyei et al., 2021) and asset prices were affected (Bossman, 2021; Bossman et al., 2022).

Information flows and spillovers are predominant in crises periods. Resultantly, due to the action(s) of rational, albeit irrational investors, any COVID-19 news item that hits the market would be reacted to, leading to the emergence of short-lived connections within and across financial markets. In the era of the COVID-19 pandemic, the number of confirmed cases of the coronavirus, proposed policy actions, retirement plans, unemployment levels, etc., are all possible factors that cause sudden decisions in financial markets (Agyei et al., 2021; Bossman, 2021; Owusu Junior et al., 2021) and, hence, could be attributed to the intensified connectedness and spillovers between Islamic and conventional stock markets. Corollary to the panic decisions, which emanate from transitory factors, rebalancing of portfolios may be ineffective in the short term.

The pandemic has stayed with us for two years and counting, and with the emergence of diverse variants of the virus, the circulation of COVID-19 related news items, both negative and positive, are expected to persist in financial markets. Therefore, the momentary spillovers between Islamic and conventional stock markets (as well as financial markets in general) are likely to be persistent in the era of the COVID-19 pandemic.

Overall, our results are suggestive that spillovers largely dominate in the short-term within high frequency/spillover bands 1 and 2 (3.14–0.79 and 0.79 to 0.20), representing the short-term. That is, the total spillovers existent across and within the Islamic and G7 stock markets could be seen to be attributable to the short-term. Comparatively, the frequency-domain results suggest that, whereas Islamic stocks are more likely to be immune to the shocks presented to financial markets globally during the COVID-19 pandemic, G7 stocks are less immune to these shocks owing to the presence of sporadic volatility clusters in the studied period. These findings are supported by the extant literature such as Balli et al. (2019), Mirz et al. (2021), Shahzad et al. (2018), and Yarovaya et al. (2021). For instance, Mirz et al. (2021) report that Islamic equities are more robust to COVID-19 shocks than non-Islamic counterparts during the pandemic's peak months, outperforming non-Islamic markets.

Further assessments of the results in Table 3 (and those in the Appendix) reveal the net transmitters and recipients of return volatilities among the markets. In the short-term, within the spillover band 3.14 to 0.79, the net transmitters of spillovers across the Islamic and G7 markets are India, Indonesia, Kuwait, Malaysia, Morocco, and UAE for the Islamic markets studied whereas except for Japan, all other G7 markets are net transmitters of shocks. Within Islamic stocks only, all the aforementioned Islamic markets, except for India, remain as net transmitters whereas Jordan and Morocco are found to be net transmitters of shocks to the studied Islamic markets at high frequencies (within band 3.14 to 0.79) only. For the G7 markets, Canada, Japan, and the USA (France, Germany, Italy, and the UK) proved to be net recipients (transmitters) of spillovers at high frequencies between 3.14 and 0.79.

In the long-term, India, Indonesia, Kazastan, Kuwait, Malaysia, Qatar, Saudi Arabia, and UAE are found to be net transmitters of spillovers across Islamic stocks, whereas all markets except for Italy and Japan are found net transmitters of shocks in G7 stocks. The findings suggest that the nature of volatility spillovers across and within Islamic and/or G7 markets is time-varying and frequency-dependent which is consistent with the HMH (Müller et al., 1993). Additionally, the findings are commensurate with the conclusion of Mensi et al. (2021) who also reveal that volatility spillovers among Islamic and conventional equities (from the BRICS markets) were contingent on time scales and frequencies. Other empirical works, such as Balli et al. (2019), Hung and Vo (2021), Shahzad et al. (2018), and Yarovaya et al. (2021), also substantiate our findings. From the findings, investors who hold assets in conventional markets – in search of competitive yields – are likely to adapt to Islamic assets in turbulent times, which is consistent with the AMH and CMH of Lo (2004) and Owusu Junior et al. (2021) respectively.

### 5.2 Robustness

Following the works of Antonakakis et al. (2020), we employ the time-varying parameter vector autoregressive (TVP-VAR) technique^7^ to confirm the robustness of our results.

With motivations from Koop and Korobilis (2014), Antonakakis et al. (2020) present a TVP-VAR connectedness technique that extends Diebold and Yilmaz's (2012, 2014) originally suggested connectedness technique by allowing the variance-covariance matrix to fluctuate using a Kalman filter estimation with forgetting factors. This approach, the TVP-VAR connectedness, gets around the problem of rolling-window sizes that are frequently picked at random. In accounting for dynamism, adaptability, and heterogeneity in assets connectedness, and examining the frequency-dependent connectedness between Islamic and conventional stocks, we inculcated rolling window analysis. Therefore, considering the relative merits of Antonakakis et al.’s (2020) TVP-VAR connectedness model, it serves as an appropriate technique to assess the robustness of our findings from the Baruník and Křehlík (2018) spillover index approach.

The plots in Figure 4 present the total connectedness index between the studied Islamic and G7 stocks (a), Islamic stocks only (b), and G7 only (c). The average dynamic connectedness indices in Table 4^8^ numerically support the results in Figure 4. Moving from left to right, the dotted lines in the plots represent significant event dates for the Chinese market crash in January 2016 (Dutt, 2016), the Brexit effect (David, 2016), the announcement of the first confirmed case of COVID-19 infection in China on 7 January 2020 (Holshue et al., 2020), and the declaration of the COVID-19 as a pandemic by the World Health Organisation on 11 March 2020, respectively. These are specified for easy identification and inference of contagious connectedness between Islamic and conventional stock markets.

**Figure 4:** Total connectedness index. (a) – between Islamic and G7 markets; (b) – between Islamic markets only; (c) – between G7 markets only.

**Table 4:** Average dynamic connectedness between Islamic and G7 stocks.

It is essential to note that the results from the TVP-VAR estimations corroborate the initial findings documented from the Baruník and Křehlík (2018) approach. Specifically, from Figure 4 (a), we find high dynamic connectedness (averaging over 40%) between Islamic and G7 stock markets and in the COVID-19 pandemic era, the connectedness increases substantially. For all event dates, we find evidence of sporadic increases in connectedness between Islamic and G7 markets. A similar observation is evident when the two markets are studied alone. Our findings divulge that among the specified significant dates, the hikes in dynamic connectedness between the studied Islamic and conventional markets are more intense in the COVID-19 era. The connectedness indices between the markets are higher in the studied COVID-19 pandemic period (2020/2021). Therefore, the contagious spillovers revealed in the BK-18 results are confirmed by the results from the TVP-VAR connectedness model.

Similar to the BK-18 results, we find that in normal (stressed) trading periods, Islamic markets are less (more) connected than conventional markets. However, this needs to be assessed in the frequency domain to ascertain the investment horizon(s) characterised by high spillovers. Consequently, we underscore the importance of the frequency-domain results from the BK-18 approach. Moreover, from the TVP-VAR model's average dynamic connectedness indices (see Table 4), we identify the sources of contagion between the studied Islamic and conventional stock markets to include UAE, Saudi Arabia, Canada, Kuwait, and Malaysia. These corroborate the results in the BK-18 approach when analysed in the frequency domain. Backed by empirical evidence, it is natural and intuitive to note that these results are further substantiated by the directional and pairwise connectedness results in Figures 5 and 6.

**Figure 5:** Net total directional connectedness.

**Figure 6:** Directional connectedness of Islamic and G7 stocks.

Overwhelming similarities in the results are offered by the BK-18 and the TVP-VAR models. As a result, we conclude that our findings are robust to new techniques that account for dynamisms in assets connectedness resulting from the heterogeneous and adaptive behaviour of market participants.

## 6 Practical implications

Generally, our results suggest that spillovers largely dominate in the short-term within high frequency/spillover bands 3.14–0.79 for both Islamic and conventional markets. That is, the total spillovers existent between Islamic and G7 stocks could be attributed to short-term transitory conditions (Jena et al., 2021). These results are consistent with the EMH such that in the short-term, asset prices fully reflect all pertinent information (Fama, 1970, 1998), resulting in exuberant market dynamics. Impliedly, investors should be wary of the high co-movement of Islamic and G7 stocks in the early trading days (up to a week) in crises periods since diversification, safe-haven, and hedging opportunities may be futile.

During turbulent trading days, speculators may have to focus on Islamic and conventional markets in the medium-to long-term horizons, where volatilities are less prevalent. More importantly, our findings divulge that diversification between Islamic and conventional equities would be viable in the medium- and long-term horizons only. Practically, in the intermediate- and long-term horizons, the EMH may not hold as international investors might have adapted and rebalanced their portfolios regarding their behavioural intentions. Investors would seek to maximise (mitigate) portfolio returns (risks) across investment horizons and, hence, should they find themselves in tumult trading periods, it is optimal that they adapt to the heterogenous market responses based on their appetite for risks. This observation is supported by the AMH, HMH, and CMH of Lo (2004), Müller et al. (1993), and Owusu Junior et al. (2021), respectively. Therefore, in the intermediate- and long-term, Islamic and conventional markets are characterised by dynamic, adaptive, and heterogeneous activities.

Stocks from the UAE, Saudi Arabia, Canada, Kuwait, and Malaysia possess high spillovers and, therefore, investors should be wary of these equities during asset allocation and portfolio construction. Individual stock markets have their market-specific shocks, which are significant and requires policymakers and international investors to consider such shocks when making respective decisions on market regulation and portfolio management. Furthermore, Islamic stocks only are less (more) connected in tranquil (turbulent) trading periods. Given the results from the directional and pairwise connectedness, investors could adjust their portfolio holdings across investment horizons. Specifically, investors and regulators must note that the pandemic has lasted for two years and counting, and we project that with the emergence of several viral strains, the circulation of COVID-19-related news items, both good and bad, would continue in financial markets. As a result, in the period of the COVID-19 outbreak, the ephemeral spillovers between Islamic and conventional stock markets (as well as financial markets in general) are expected to endure. These factors must be considered in the regulation of financial markets as well as in asset allocation and portfolio management.

## 7 Conclusions

This study utilised the Baruník and Křehlík (2018) (BK-18) spillover index to examine the dynamic connectedness and spillovers between Islamic and conventional stock markets to reveal the time- and frequency-domain dynamics of the two asset classes during different market conditions. The daily stock market indices spanning between 23 November 2015 and 08 September 2021 for 17 key Islamic markets (Bahrain, Bangladesh, India, Malaysia, Indonesia, Kazastan, Pakistan, Egypt, Iraq, Jordan, Kuwait, Oman, Palestine, Qatar, Saudi Arabia, UAE, and Morocco) and G7 economies (Canada, France, Germany, Italy, Japan, UK, and the USA) were employed in the processing and analysis. Specifically, we investigate: whether the fundamental relationship between Islamic and conventional stocks remains the same in the COVID-19 era; the extent to which stocks from Islamic and conventional markets are connected in stress periods; whether the connectedness between Islamic and conventional stocks differ across investment horizons; whether the connectedness between Islamic and conventional markets evolve from interdependence or contagion, and which markets transmit or receive the most shocks among Islamic and conventional markets.

Through the BK-18 framework, we found that spillovers in the very short-term (intraweek) are comparatively higher than in the medium-to long-term horizons, implying that all the markets respond quickly to shocks in the first few trading days. Thus, consistent with the EMH of Fama (1970, 1998), the Islamic and conventional markets studied are more responsive to market shocks than in later days. We conclude that short-term spillovers are more significant than intermediate-term spillovers for Islamic and conventional (G7) markets. The largest contributors of shocks to the Islamic and G7 markets are France, UAE, and Malaysia in the high-frequency bands (i.e., short-term), notably in the first spillover band (3.14–0.79, corresponding to 1–4 trading days). Canada, Kuwait, and Saudi Arabia are found to be the largest contributors of shocks to the selected Islamic and G7 stock markets in medium- and long-term periods, with Iraq being both the least contributor and recipient of shocks between the markets studied. Saudi Arabia and Malaysia were found to be the largest recipient of spillovers in the short-term and intermediate-to long-term periods respectively.

In addition, during the COVID-19 period, whereas spillovers across Islamic markets are relatively stable, the spillovers are more observable and intensified in G7 stocks especially in the short-term across spillover bands 1 and 2 (intraweek and week-to-fortnight). We, thus, conclude that during market turbulences, conventional stocks are prone to more volatilities than Islamic stocks. Furthermore, from our findings, we suggest that the nature of volatility spillovers across and within Islamic and/or G7 markets is time-varying and frequency-dependent which is consistent with the HMH of Müller et al. (1993), the AMH of Lo (2004) and the CMH of Owusu Junior et al. (2021). Our conclusions are backed by the literature such as Balli et al. (2019), Fassas (2020), Haddad et al. (2020), Liu et al. (2021) Mensi et al. (2021), Mirz et al. (2021), Shahzad et al. (2018), and Yarovaya et al. (2021). More importantly, we infer incidences of financial contagion (in line with Forbes and Rigobon, 2001, 2002) – evidenced by increases in spillovers – within 2017/18 and 2020/21 which are attributable to the Brexit and COVID-19 pandemic respectively and substantiates the delayed contagion hypothesis presented by Boako and Alagidede (2017). Thus, we report significant contagious spillovers in the COVID-19 era, which corroborate those in the recent studies (viz., Akhtaruzzaman et al., 2021; Fassas, 2020; Haddad et al., 2020; Hung and Vo, 2021; Liu et al., 2021; Papadamou et al., 2021) which examine financial contagion in the COVID-19 era.

Investors and governments will benefit greatly from our findings. Spillovers are time-varying, and asymmetric, which should be kept in mind by equity investors. Specifically, amid financial and health crises, investors may utilise knowledge about market patterns and volatility to hedge their positions against lower stock returns, especially in the near term (up to four trading days), when spillover is more intense. According to the HMH and CMH, equity investors may change their investment strategy owing to heterogeneous occurrences. Regardless of the time horizon, Islamic stocks provide diversification benefits relative to the G7 stocks. When forecasting stock price volatility and constructing equity portfolios, portfolio managers should not disregard the information on policy amendments resulting from market shocks like the COVID-19 pandemic. During financial turmoil, policymakers should pay close attention to spillovers, since they undermine cross-market connections.

Equity fund and/or portfolio managers and policymakers could forecast the impact of their policies and reforms by using data on frequency dynamic spillover intensities and directions. Rebalancing portfolios may be unproductive in the near run of the COVID-19 pandemic, as a corollary to panic judgments based on transient factors. Given the results from the directional and pairwise connectedness, knowledge about the dynamic interrelations across different time scales or investment horizons is essential to arrive at optimal asset management (Salisu et al., 2020). Timely rebalancing of portfolios, on the part of international investors and/or portfolio managers, is essential to benefit from the diversification, safe haven, and hedge opportunities between Islamic and conventional stocks. Similarly, to attract international flows through financial markets, timely interventions, which result from optimal forecasts of policy impacts on financial markets, by regulators are essential to curtailing the ‘own’ market shocks suffered by financial markets and to a large extent, minimise the total shocks available to financial markets.

## Declarations

### Author contribution statement

Ahmed Bossman: Conceived and designed the experiments; Analyzed and interpreted the data; Wrote the paper.

Peterson Owusu Junior, Aviral Kumar Tiwari: Conceived and designed the experiments; Analyzed and interpreted the data; Contributed reagents, materials, analysis tools or data.

### Funding statement

This research did not receive any specific grant from funding agencies in the public, commercial, or not-for-profit sectors.

### Data availability statement

Data included in article/supplementary material/referenced in article.

Stock indices for all the countries were retrieved from EquityRT and are available at https://equityrtcom/.

### Declaration of interests statement

The authors declare no conflict of interest.

### Additional information

No additional information is available for this paper.

## Appendix A Supplementary data

Volatility_Spillover_Isl_Con_Stocks_Supplementary_File Volatility_Spillover_Isl_Con_Stocks_Supplementary_File

## Footnotes

1 Contagion may arise from any significant rise in cross-market relationships following a shock in either one country (market) or a group of countries (markets). The implication is that if there exists a co-movement between two markets during average market conditions, there is interdependence (no contagion) if the co-movement between them persists after one of them has witnessed a shock – it is contagion (or “shift-contagion”) only if there is a significant increase in an already existing cross-market relationship (Forbes and Rigobon, 2001, 2002). For extended highlights on contagion, see Forbes and Rigobon (2001, 2002), Owusu Junior et al., 2020a, Owusu Junior et al., 2020b, Owusu Junior et al., 2020c, etc.

2 According to Baruník and Křehlík (2018), the generalised causation spectrum is the squared modulus of the weighted complex numbers, resulting in a real-valued quantity.

3 As seen in Eqs. (5, 11, and 12), the scaling factor is 100. In the practical application of the connectedness in the BK-18 framework, it is also the minimal forecast horizon H.

4 In no particular order.

5 In ascending order per country spellings.

6 The numerical indices that accompany the plots in Panels B and C can be found in the Appendix.

7 Antonakakis et al. (2020) present comprehensive notes on the TVP-VAR methodology.

8 The TVP-VAR spillover tables for the separate markets are supplied in the Appendix (Tables S6 and S7).
